# The Application of Statistical Parametric Mapping to Evaluate Differences in Topspin Backhand between Chinese and Polish Female Table Tennis Players

**DOI:** 10.1155/2021/5555874

**Published:** 2021-07-14

**Authors:** Ziemowit Bańkosz, Sławomir Winiarski

**Affiliations:** Department of Biomechanics, Faculty of Physical Education and Sports, University School of Physical Education in Wroclaw, Poland

## Abstract

The research is aimed at comparing the kinematics (the movement pattern in the most important joints and accelerations of the playing hand) between female table tennis players coached in Poland (POL) and China (CHIN) during the performance of a topspin backhand stroke (so-called quick topspin). The study involved six female table tennis players at a high sports skill level, playing in Poland's highest league. Three were national team members of Poland (age: 20.3 ± 1.9), while the other three were players from China (age: 20.0 ± 0.0). Kinematics was measured using MR3 myoMuscle Master Edition system—inertial measurement unit (IMU) system. The participants performed one task of topspin backhand as a response to a topspin ball, repeated 15 times. Statistical parametric mapping (SPM) was calculated using SPM1D in a Python package that offered a high-level interface to SPM1D. The SPM method allowed for the determination of differences between the Chinese and Polish female athletes. The differences found are probably mainly due to differences in the training methodologies caused by different coaching systems. The observed differences include, among others, greater use of the so-called small steps in order to adapt and be ready during the back to ready position and backswing phases, which gives the CHIN players slightly better conditions for preparation for the next plays. The CHIN players' position compared to that of the POL players favours a quicker transition from the backhand to the forehand play. This difference is probably related to the difference in the dominant playing styles of the groups studied. Despite the differences in movement patterns in both groups, the exact value of playing hand was achieved. This may be a manifestation of the phenomenon of equifinality and compensation. All the differences found are probably mainly due to differences in the training methodologies caused by different coaching systems.

## 1. Introduction

As a very complex and multifaceted sport, table tennis is characterized by various strokes, legwork techniques, tactical solutions and playing styles, and a multitude of solutions for an almost infinite number of game situations. The main groups of strokes that yield points are topspin strokes, introduced to the game in the 1950s by Japanese players [1]. Players use many variations of topspin strokes in their game (e.g., backhand and forehand strokes, differing in strength involved, speed of ball rotation, flight trajectory, ball speed, and the moment of hitting the ball) depending on the solution used or the need to adjust to ball parameters. Table tennis players must also adjust their position to the ball using a different kind of footwork, changing kinematics and kinetics characteristics of body segments [2, 3]. These differences lead to a large variety and variability of movement in this sport. Issues related to movement variability have recently been quite often addressed in the literature. Traditionally, movement variability is considered to reflect the “noise” in the system of human movements, while learning a given activity requires decreasing variability as it is perceived as incorrect [4, 5]. Movement variability is also viewed and considered a normal phenomenon, resulting from the diversity and variability present in the entire biological system used by humans, and its occurrence is associated with adaptive and functional processes [6]. Movement variability has been explained using many theories available in the literature, such as generalized motor program [7, 8], GMP-uncontrolled manifold (UCM) [9], and dynamic systems theory [5]. Assessing the occurrence and scale of movement variability appears to be extremely important in the sports training process. It seems to be also critical in the process of improving skills of purposive movements and explaining how to control human movements. Linear measures have been used in the assessment of variability, such as standard deviation, range, or coefficient of variation. Taking into account discrete (numerical) or serial data, i.e., continuous and changing over time, would improve the assessment of variability. This is because when assessing movement coordination, for instance, the change of the angle in a given joint over time, and comparing the repetitions by one or many people, a method should be used to compare time waveforms rather than just single, selected parameters. Such criteria are met by the statistical parametric mapping (SPM) method. It is the gold standard statistical method dedicated to numerical signal data analysis. For the one-dimensional variables recorded with the motion analysis system, the general SPM model can be simplified to the one-dimensional model SPM1D. This method and its characterization were presented in previous studies [10].

The assessment of variability of movement seems to be important in table tennis, which is a very complex sport, where technique and its improvement are the essential elements used to achieve the champion level, with the basis of the technique being a stroke and precise hitting the ball with the racket. The few available studies on table tennis and the variability of movement have been based on the methods of evaluation of standard deviation, correlation, and analysis of variance (ANOVA and least significant difference (LSD)) and presented UCM calculations. Iino et al. emphasized that the possibility of using different configurations in the evaluated joints to stabilize the vertical angle of the racket in table tennis strokes can be a critical factor in playing performance [11]. A previous study by Bańkosz and Winiarski also evaluated the variability of movement by analyzing the coefficient of variation of kinematic parameters in selected important moments of the hitting movement [10, 12]. However, the coordination of movements in individual joints was taken into account to a small extent. The variability of temporal and spatial coordination of movements, the possibility of compensation, and functional variability are significant problems in the coaching practice and in the process of teaching and improving technique and its monitoring. Making the coaches and players aware of the different variants of strokes even for a specific solution (e.g., playing with the right strength, speed, and rotation to the same place) seems to be very important and necessary for improving the training process. Therefore, copying and imposing a single pattern of performing the movement seem to be a wrong way. Considering the differences between athletes and looking for individual technical solutions instead would be a better choice [10].

Interpersonal variation of the sports technique may result, for example, from gender differences, differences in anatomical structure, and differences in sports skill level. The diversity of techniques due to the training system also seems to be an interesting issue. Identification of differences and, at the same time, similar or perhaps unchangeable elements of table tennis stroke techniques in athletes coached using different training systems can provide important insights into the technique of performing a given stroke. Some differences in the technique may indicate the possibility of using different solutions in the performance of the stroke, while the same, similar, and unchanging elements may highlight their importance in table tennis. Therefore, the aim of the research was to compare the kinematics between female players coached in Europe (Poland) and Asia (China) during the performance of a topspin backhand stroke. In accordance with the findings of other authors and previous studies [12, 13], it was assumed that, despite the comparable level of players, there are many differences in the kinematics of topspin backhand between them. The greater differences between the players would occur in the joints and segments located farther from the place of the racket contact with the ball (upper body and shoulder joint) than in those closer, located in the playing hand (wrist joint). It can also be assumed that at the key instant of the stroke, which is the moment of maximum acceleration, occurring at around the contact between the racket and the ball, the least differences are observed in players' kinematics.

## 2. Material and Methods

### 2.1. Study Design

It was an observational study with adopted retrospective convenience sampling. The minimal sample size of our data was determined in the planning stage of the experiment using the margin of error approach to get results as accurate as needed (with an assumed 5% margin of error at 95% level of confidence and *α* level of 0.05). The assumed standard deviation was taken from preliminary studies using the same population of interest.

### 2.2. Participants

The study involved six female table tennis players at a high sports skill level, playing in the highest league in Poland (Ekstraklasa table tennis league). Three of them were national team members of Poland (POL) in the category of adult players (age: 20.3 ± 1.9 y.), while the other three were players from China (CHIN, age: 20.0 ± 0.0 y.), coached within the Chinese training system (i.e., in China). All of the players had more than 10 years of experience in table tennis and presented the offensive style of the game. One player from China was a left hander. Average body height was 161.7 ± 4.5 cm in the group of Polish players and 162.7 ± 4.1 cm in the group of Chinese players, whereas body weight was 59.0 ± 6.9 kg and 56.7 ± 6.4 kg, respectively.

Before the study, all participants were informed about the purpose of the study and the possibility of withdrawing participation at any stage, without giving a reason. All the participants provided informed consent before the research. Pain or recent injury was the exclusion criterion for the study participants. All procedures performed in this study received positive approval from the Senate's Research Bioethics Commission at the University School of Physical Education in Wrocław, Poland (Ethics IRB number 34/2019).

### 2.3. Laboratory Set-Up

Kinematics was measured using the MR3 myoMuscle Master Edition system (myoMOTION™, Noraxon, USA, Figure 1). The myoMOTION system consists of a set of (1 to 16) sensors using inertial sensor technology. Based on the so-called fusion algorithms, the information from a 3D accelerometer, gyroscope, and magnetometer is used to measure the 3D rotation angles of each sensor in absolute space (yaw-pitch-roll, also called orientation or navigation angles, [12]). Inertial sensors were located on the body of the study participant to record the accelerations, according to the myoMOTION protocol described in the manual. The accuracy and validity of the inertial measurement unit (IMU) system in angle determination were the subject of the previous research [14, 15].

Sensors were attached with elastic straps and self-adhesive tape. The sensors were placed bilaterally so that the positive *x*-coordinate on the sensor label corresponded to a superior orientation for the trunk, head, and pelvis (Figure 1). For the limb segment sensors, the positive *x*-coordinate corresponded to a proximal orientation. For the foot sensor, the *x*-coordinate was directed distally (to the toes). At the beginning of the measurement, each participant was checked and the system was calibrated according to the manufacturer's recommendations. The recording speed of the piezoelectric sensor was adjusted to the maximal sampling rate for a given sensor (100 Hz per sensor) for the whole 16-sensor set. Noraxon's IMU technology mathematically combines and filters incoming source signals on the sensor level and transmits the 4 quaternions of each sensor. We used system-built fusion algorithms and Kalman filtering (digital bandpass finite impulse response filter (FIR)). This mode allowed direct access to all unprocessed raw IMU sensor data.

### 2.4. Experimental Procedures

The participants performed one task of topspin backhand (TBH) as a response to a topspin ball, repeated 15 times. Each player was asked to hit the ball in the early stage of its flight (so-called quick topspin) and to reach the marked area in the corner of the table (30 × 30 cm) diagonally (after instruction: “play diagonally, accurately, and as quick as you can”). After video analysis, only successful shot considered “on table” and played diagonally was recorded for further calculations (missed balls, balls hit out of bounds, and balls hit into the net were excluded). The balls were shot by a dedicated table tennis robot (Newgy Robo-Pong Robot 2050, Newgy Industries, Tennessee, USA, Figure 1) at constant parameters of rotation, speed, direction, and flight trajectory. The settings of the robot were as follows:

- Rotation type: topspin
- Speed (determines both speed and spin, where 0 is the minimum and 30 is the maximum): 18
- Left position (leftmost position to which the ball is delivered): 15
- Wing (robot's head angle indicator): 7.5
- Frequency (time interval between balls thrown): 1.4 s

Each player had had three to five familiarization trials before the task. The same racket with the following characteristics was used for the experiment: blade, Jonyer-H-AN (Butterfly, Japan); rubber, Tenergy 05, 2.1 mm (Butterfly, Japan); Plastic Andro Speedball 3S 40+ balls (Andro, Germany); and a Stiga Premium Compact table (Stiga, Sweden).

### 2.5. Kinematics

A total of 90 cycles of topspin backhand stroke were studied. Based on the ISB recommendations concerning the definitions of the joint coordinate system of various joints for the reporting of human joint motion [16, 17], the following angles (measured in degrees) were chosen for both sides and sampled every 0.01 percent of cycle time:

- Ankle dorsiflexion/plantar flexion (AFE): rotation of the foot with respect to the tibia coordinate system in the sagittal plane; a negative sign denotes plantar flexion (extension) and positive sign dorsiflexion (flexion)
- Ankle abduction-adduction: movement of the foot away or towards the midline of the body; a negative sign denotes adduction while positive sign abduction
- Ankle inversion-eversion: rotation of the foot around its long axis; a negative sign denotes eversion (away from the median plane) while positive sign inversion (towards the median plane)
- Knee flexion-extension (KFE): movement of the tibia with respect to the femur coordinate system in the sagittal plane; a negative sign denotes extension and positive flexion
- Hip flexion-extension (HFE): movement of the femur with respect to the pelvis coordinate system in the sagittal plane; a negative sign denotes extension while positive flexion
- Hip abduction-adduction (HAA): movement of the femur with respect to the pelvis coordinate system in the frontal plane; a negative sign denotes adduction while positive abduction
- Hip internal-external rotation (HIER): internal or external movement of the femur with respect to the pelvis coordinate system in the transversal plane; a negative sign denotes internal while positive external rotation
- Lumbar internal-external rotation (LIER): internal or external movement of the loins in the transversal plane; a negative sign denotes internal while positive external rotation
- Thoracic internal-external rotation (ThIER): internal or external movement of the thorax relative to global coordination system in the transversal plane; a negative sign denotes internal while positive external rotation

For the upper extremity (playing side), a simplified biomechanical model was adopted based on the predominant plane of movement as described by Wu et al. [17] with segments of interest being the thorax, clavicle, scapula, humerus, forearm, and carpus of the hand. Based on the adopted sequence of Euler angles, the following angles were computed:

- Shoulder flexion-extension (ShFE): movement of the humerus relative to the thorax in sagittal plane; negative sign denotes extension while positive flexion
- Shoulder abduction-adduction (ShAA): movement of the humerus relative to the thorax in the frontal plane; negative sign denotes adduction while positive abduction
- Shoulder internal-external rotation (ShIER): movement of the humerus relative to the thorax in the transversal plane; a negative sign denotes internal (medial) while positive external (lateral) rotation
- Elbow flexion-extension (EFE): movement of the forearm relative to the humerus along the transversal axis; negative sign denotes (hyper)extension while positive flexion
- Wrist flexion-extension (WFE): movement of wrist relative to the radius along the transversal axis and measured between upper arm and hand sensors; a negative sign denotes extension while positive flexion
- Wrist supination-pronation (WSup): movement of wrist relative to the radius along the axis and measured between the upper arm and hand sensors; pronation is a positive rotation and supination is a negative rotation
- Wrist radial abduction-adduction (WRad): movement of wrist relative to the radius and measured between the upper arm and hand sensors; adduction (or ulnar deviation) is negative while abduction (or radial deviation) is positive

The movement of the playing hand was used to assess specific events of the cycle:

- Ready position, where the hand is not moving after the previous stroke, just before the swing
- Backswing, which is the moment when the hand changes direction from backward to forward in the sagittal plane after the swing
- Accmax, which is the moment of maximum acceleration of the hand and the moment when the hand reaches the maximum acceleration
- Forward, which is the moment when the hand changes the direction from forward to backward in the sagittal plane after the stroke (the end of the cycle and the beginning of the next cycle)

The phases between defined events were as follows: back to ready position phase (between the forward and ready position), backswing phase (between ready position and backswing), hitting phase (between backswing and Accmax), and forward end phase (between Accmax and forward). The timing of events was analyzed and compared between the POL and CHIN players.

### 2.6. Statistical Analysis

Statistical calculations were performed using Statistica 13.1 (TIBCO Software Inc.). The sample size was estimated using recommendations postulated by Kontaxis et al. [18]. The statistical power was sufficient to detect the described differences. Power analysis of discrete data was performed to estimate the SPM test power. For the extracted data and for the significant changes (alpha = 0.05), the partial *η*^2^ effect size was found between 0.62 and 0.86. The SPM test was applied to identify the differences between groups in the movement patterns in individual joints and changes in the acceleration of the playing hand. The SPM was calculated using SPM1D in a Python package that offers a high-level interface to SPM1D. Angle-time numerical series were averaged over trials and reported against cycle time (Figure 2(a)). For each participant and selected time-dependent angular numerical data, a two-sample *t*-test SPM{*t*} function (with alpha = 0.05, nonsphericity correction, and assumption of unequal variances) was numerically computed to check the level of similarity between the movements [19, 20]. For each test, a statistical parametric map SPM{*t*} (Figure 2(b)) was created by calculating the conventional univariate *t*-statistic at each point of the gait curve [21–24]. When an SPM{*t*} crossed the assumed threshold, an additional threshold cluster was created, indicating a significant difference (a grey area) between two compared joint motion patterns in a specific location of the gait cycle. In the present study, because of the high number of statistical analyses, the SPM results are visualized in a summarised manner. Instead of SPM{*t*} curves, blue bars are shown, indicating the significance during the cycle (Figure 2(c)).

## 3. Results and Discussion

The study is aimed at evaluating the differences in movement kinematics using the SPM method between two different groups of female table tennis players. The application of the SPM test allowed for the identification of the differences between groups in the movement patterns in individual joints and changes in the acceleration of the playing hand. The basic difference that can be noticed is the time of occurrence of the beginnings and ends of the individual movement phases. For the POL players, the backswing phase starts slightly earlier (about 46% of the cycle duration for POL, 54% for CHIN players) similarly to the hitting phase (83% and 87%, respectively), whereas the average time of the maximum hand acceleration (Accmax) is very similar for both groups (about 96% of the cycle duration). The observation and description of the way of coordinating the movements when hitting the backhand topspin reveals that the average movement pattern (changes in joint angles throughout the cycle) is consistent with that described in previous studies [25, 26]. The following movements were observed in the backswing phase: lower limb flexion, upper body flexion (forward bend), adduction and internal rotation in the shoulder joint, elbow joint flexion, and flexion, pronation, and palmar flexion in the wrist joint. In the hitting phase (with different time of inclusion of individual segments into the movement, according to the principle of the proximal-to-distal movement sequence), the following movements were observed: extension in the lower limb and upper body joints, abduction, flexion, and external rotation in the shoulder joint, extension and supination in the elbow joint, and extension, supination, and radial abduction in the wrist joint.

The analysis of the SPM test results allowed for the observation of the differences in the movement patterns in the individual analyzed joints.

1. Ankle joints: the movement pattern in the ankle joints is characterized by the occurrence of many periods that differ between the two groups studied. The lack of differences in the flexion-extension movement (dorsiflexion, Figure 3) in the nonplaying side ankle joint (i.e., throughout the hitting phase) and wave-like changes in ankle joint movement observed with higher frequency in CHIN female athletes (Figure 3) are noticeable
2. Knee joints: in the flexion-extension movement of the knee joints, the wave-like character of the changes in the back to ready position phase and the backswing phase observed in CHIN is noteworthy. Significantly, more periods differing between the two groups occur in the right knee joint (Figure 3), in which the average flexion range is larger in POL compared to the CHIN group during the entire cycle
3. Hip joints: in hip joint movements, there are more periods of differences concerning the right hip joint. CHIN players exhibit greater abduction and external rotation throughout the cycle in the right hip joint. It is noteworthy that there were no differences between the groups in the significant part of the backswing phase in the abduction movement in the nonplaying side hip joint and the part of the backswing and hitting phases in the rotation movement in these joints (Figure 3).
4. Joints of the upper body: very few differences were observed in the flexion-extension movements in the lumbar region, in which flexion can be observed in the backswing phase and extension was found in the hitting phase (Figure 4). The range of rotation movement was slight (about 5 deg), more pronounced in CHIN, whereas in the POL group, it was characterized by high variability (high SD value throughout the cycle). The movement of the upper body (thoracic region) differentiates the two groups the most in the sagittal plane (flexion-extension). In CHIN players, this movement is used to a greater extent (about 30-40 deg), from slow flexion in the backswing phase, through faster flexion in the initial hitting phase, to the extension in the Accmax region and later (Figure 4). The rotation of this part of the upper body and lateral flexion in the backswing phase and most of the hitting phase does not show differences between the two groups. These movements take place in small ranges of several degrees
5. Shoulder joint of the playing limb: in the shoulder joint of the playing limb, it can be observed that the differences mainly concern the back to ready position phase in all planes (Figure 5). In the flexion-extension movement, differences also occur at the end of the forward phase. Greater abduction and external rotation can be also observed in the part of the backswing and hitting phases in the discussed joints in the CHIN female players (Figure 5). It should also be emphasized that there is a period with no differences in the flexion-extension movement in a significant part of the backswing and hitting phases (up to the moment of reaching the maximum acceleration—Accmax)
6. Elbow joint of the playing limb: the SPM test revealed differences in flexion-extension movement at the elbow joints in the major part of the back to ready position phase, part of the backswing phase, and the end of the hitting phase (Figure 5). Nevertheless, both groups showed elbow flexion in the backswing joint in the back to ready position phase (up to circa 70-90 deg), maintaining this flexion or very slow extension during the backswing phase, and quite a rapid extension during the hitting phase (up to circa 20-40 deg)
7. Wrist joint of the playing limb: the fewest periods of differences between the two groups demonstrated by the SPM test occur in the movement of elbow flexion and radial abduction in the wrist joint (Figure 5). Maintaining the elbow flexion up to circa -20 to -30 deg can be observed in both groups in the back to ready position and backswing phases, and then, after the beginning of the hitting phase, quite a rapid movement towards radial flexion (up to circa -10-0 deg) was found. The maximum of radial flexion occurs at around Accmax, and there is a brief moment of differences between the groups during this period. The supination-pronation movement in the described joint differentiates between the two groups more. A period of no differences between the groups occurs in the back to ready position phase (from circa 5% to circa 30% of the cycle time) and in circa 91-93% of the cycle time in the hitting phase. Polish female players are characterized by using a greater range of this movement. The supination movement is rapid during the hitting phase, from the moment after the beginning of this phase to the moment of Accmax in both groups. In the extension-flexion movement in the wrist joint, it is noticeable that there are no differences in the back to ready position phase and before the Accmax moment. There is a slow flexion of the limb in the described joint in both groups during the back to ready position and backswing phases, accelerating during the hitting phase. At circa 90% of the cycle, the direction of movement changes to the extension (within circa 10 deg in both groups) at a high rate until reaching Accmax. The latter short period shows no differences between the groups

The observation that comes to mind is the occurrence of the longest periods of differentiation between the groups studied in the lower limb joints, which indicates their different use by both groups of female players. Undoubtedly, a wave-like movement in the ankle and knee joints is more pronounced in CHIN players, which reflects the use of the so-called small steps, mainly in the back to ready position and backswing phases. These steps are used to adapt to the next stroke and keep the lower limbs in constant readiness. Therefore, it can be concluded that CHIN players use these steps more often than POL and perhaps this is due to differences in coaching. Differences can be observed in the ankle joints in all planes, and they affect the entire backswing and forward phases. It is noticeable that the directions of movement in the hitting phase are the same in both groups in the ankle joints, and the differences are in the degree values. The nonplaying side ankle joint in both groups in the forward phase shows no differences and the toe-raise movement (decreasing dorsiflexion, transitioning to plantar flexion), in an approximately 20-degree range. A similar movement, but differentiating between the two groups, can be observed in the right ankle joint. For both joints, the range of motion is smaller in CHIN player. The direction of this movement in the forward phase indicates the use of upward and forward transfer of the center of gravity as an action to support the hitting movement performed by the player. The importance of this movement while performing a stroke has been highlighted in the literature [26, 27]. Wang et al. also pointed out the differences between players at different sport skill levels in the performance of movements in the joints of the lower limbs, emphasizing that these movements can be used better by an economical work with simultaneous use of the energy generated by the elastic components of the joints and muscles (based on the stretch-shortening principle) [28]. Perhaps the differences in the movement in the ankle joints shown in this paper are related to this method. As mentioned above, a wave-like movement in CHIN players was reported in flexion-extension movements in the knee joints, indicating the use of small steps in the preparation phases (back to ready position, backswing). A greater flexion angle in the right knee joint was also observed in the POL group throughout the cycle. This is probably due to the transfer of center of gravity to the right leg, emphasized more in the POL group throughout the cycle. It can be assumed that this difference allows the CHIN players to switch to forehand play faster and more flexibly after performing a pivot and is probably due to the different playing styles prevalent in the two groups. In all players, the forward phase is accompanied by the extension of the knee joints within a range of several dozen degrees. The above findings provide helpful information for coaches and players with regard to the backhand topspin technique and its modifications regarding lower limb movements.

The movement in the hip joint showed long periods of differences between the groups studied. However, similar movement directions were found in individual phases in both groups. The small rotation range of a few degrees in the hip joints should be emphasized, which, according to many authors, greatly helps generate the stroke force and high racket speed in table tennis [26–29]. It is directly suggested that the range of this movement and its use differentiates between players of different sports skill levels. The lower use of rotation in these joints is related to the type of stroke analyzed in this study. It is a topspin backhand played early against a topspin ball, so it is a counterstroke from the group of strokes that utilize the energy of the flying ball and therefore does not require the involvement of great strength of the player. Similar aspects were pointed out by Marsan et al., who evaluated the mechanical energy generated from the hip joint during different variations of strokes, finding that backhand drive required the lowest hip mechanical work [30].

In the lumbar spine, the least differences were found in the flexion-extension motion. In the backswing phase, this is a few degrees of flexion, whereas in the hitting phase-extension in both groups. The lateral flexion movement indicates that the POL players are slightly leaning to the right, with the body weight shifted to the right lower limb, again indicating a more backhanded position than in the Chinese players. The CHIN players seem to stand more universally, with the ability to transition more easily from the backhand to the forehand playing, as discussed above. The CHIN players also use a certain amount of rotation in the lumbar region during the hitting phase in contrast to POL players, who hardly use any rotation in this body segment. It must be admitted, however, that the SD values in the POL group are high, indicating great variation in the way this segment is used in the topspin backhand stroke. Nevertheless, the small range of rotation (similar in both groups) in body trunk confirms previous observations concerning the small contribution of hip and trunk rotation resulting from the type of stroke assessed.

Regarding the playing upper hand, the most differences were found in the abduction-adduction of the shoulder, flexion-extension at the elbow joint, and supination-pronation at the wrist joint. In these three cases, the differences between the groups concern much of the back to ready position phase, the beginning of the backswing, and the end of the forward phase. Actually, the end of the forward phase (from Accmax to the end of this phase) differentiates between the groups in each movement in the joints of the playing upper limb. It must be admitted, however, that the directions of movements are very similar (the curves of the graphs have a very similar shape), and the differences demonstrated in the SPM test may be due to the different times beginning the individual phases in the groups. The SPM test showed no differences in flexion-extension and external-internal rotation in the shoulder joint, in radial abduction-adduction, and flexion-extension at the wrist joint during the second part of the backswing and the beginning of the hitting phase. Movement coordination in the female players studied is consistent with that reported in the literature [25, 29]. Furthermore, the description of basic movement, presented in our work, can provide more clarity in understanding the topspin backhand technique.

The values of hand acceleration and its changes over time demonstrated in the SPM test differentiate between the groups studied for most of the cycle and in all phases, with short exceptions of ca. 20% and 40%, and in the hitting phase, especially after reaching Accmax (Figure 6).

For most of the back to ready position phase and the backswing phase, the acceleration values are close to 0. After circa half of the backswing phase, acceleration values increase until they reach maximum values at the end of the forward phase, which are very similar in both groups (about 90 m/s^2^). The pattern of acceleration values is then interesting. It is different for both groups in each phase, but it is similar at the Accmax point, and the maximum values obtained by both groups are also similar. Therefore, it can be concluded that despite the indicated differences in movement patterns in both groups, the same value of Accmax was achieved. This may be a manifestation of the phenomenon of equifinality and compensation, indicated in the literature as typical of dynamic systems and variability of movement [5, 10, 31]. Obviously, it should be added that just achieving the right amount of hand acceleration does not determine the accuracy of the play; the hitting angle, the direction of movement, and other factors are also important [32].

### 3.1. Limitations of the Study

Undoubtedly, from the standpoint of statistical calculations, the number of participants may seem to be a limitation of the study. It should be remembered, however, that the averaging of movement patterns (changes in joint angles over time) can lead to unavoidable errors in the observation of the activity of the human movement system, in which variability, differentiation, and compensation are normal and commonly occurring phenomena [5]. It should also be noted that the observations presented in this study concerned only women and one type of stroke; thus, generalization of the results should be made with caution.

## 4. Conclusions

The examinations carried out in this study allowed for a detailed description of the technique of performing a fast topspin backhand stroke, thus providing valuable information for table tennis coaches and players. The SPM method allowed for the determination of differences between the Chinese and Polish female athletes. The observed differences include, among others, greater use of the so-called small steps in order to adapt and be ready during the back to ready position and backswing phases, which gives the CHIN players slightly better conditions for preparation for the next plays. The position of the CHIN players compared to that of the POL players favours a quicker transition from the backhand to the forehand play. This difference is probably related to the difference in the dominant playing styles of the groups studied. The differences found are probably mainly due to differences in the training methodologies caused by different coaching systems. It can be also concluded that despite the indicated differences in movement patterns in both groups, the same value of Accmax was achieved. This may be a manifestation of the phenomenon of variability of movement, as well as equifinality and compensation.

## Figures and Tables

**Figure 1:** Measurement site.

**Figure 2:** SPM procedure. The SPM, like other statistical methods, has assumptions. The assumptions for the SPM{*t*} paired sample *t*-test include continuous waveforms with an equal sample rate and a number of data points; the sample size (or data set size) should be greater than 5 in each group; each waveform should come from a random sample and be normally distributed over time; the waveforms of interest should be spread similarly between the two groups (homogeneity of variance that is maintained over time).

**Figure 3:** Lower extremity kinematics. Red line: average values of POL; green line: average values of CHIN; grey areas: SD values. Blue bars indicate the significance during the cycle.

**Figure 4:** Torso kinematics. Red line: average values of POL; green line: average values of CHIN; grey areas: SD values. Blue bars indicate the significance during the cycle.

**Figure 5:** Upper extremity kinematics. Red line: average values of POL; green line: average values of CHIN; grey areas: SD values. Blue bars indicate the significance during the cycle.

**Figure 6:** Hand acceleration. Red line: average values of POL; green line: average values of CHIN; grey areas: SD values. Blue bars indicate the significance during the cycle.

## Data Availability

The supplementary data (containing angle waveforms and accelerations) used to support the findings of this study are included within the supplementary materials.

## Supplementary Materials

Supplementary Materials Angles and accelerations.

## References

[1] Fuchs M., Liu R., Malagoli Lanzoni I. (2018). Table tennis match analysis: a review. *Journal of Sports Sciences*.

[2] Malagoli Lanzoni I., Bartolomei S., Di Michele R., Fantozzi S. (2018). A kinematic comparison between long-line and cross-court top spin forehand in competitive table tennis players. *Journal of Sports Sciences*.

[3] Shao S., Yu C., Ugbolue U., Malagoli Lanzoni I., Baker J., Gu Y. (2020). Mechanical character of lower limb for table tennis cross step maneuver. *International Journal of Sports Sciences & Coaching*.

[4] Bartlett R., Wheat J., Robins M. (2007). Is movement variability important for sports biomechanists?. *Sports Biomechanics*.

[5] Stergiou N., Decker L. M. (2011). Human movement variability, nonlinear dynamics, and pathology: is there a connection?. *Hum Mov Sci*.

[6] Stergiou N., Yu Y., Kyvelidou A. (2013). A perspective on human movement variability with applications in infancy motor development. *Kinesiology Review*.

[7] Schmidt R. A. (2003). Motor schema theory after 27 years: reflections and implications for a new theory. *Research Quarterly for Exercise and Sport*.

[8] Summers J. J., Anson J. G. (2009). Current status of the motor program: revisited. *Human Movement Science.*.

[9] Scholz J., Schöner G. Use of the uncontrolled manifold (UCM) approach to understand motor variability, motor equivalence, and self-motion.

[10] Bańkosz Z., Winiarski S. (2020). Statistical parametric mapping reveals subtle gender differences in angular movements in table tennis topspin backhand. *International Journal of Environmental Research and Public Health*.

[11] Iino Y., Yoshioka S., Fukashiro S. (2017). Uncontrolled manifold analysis of joint angle variability during table tennis forehand. *Human Movement Science*.

[12] Bańkosz Z., Winiarski S. (2020). Kinematic parameters of topspin forehand in table tennis and their inter- and intra-individual variability. *Journal of Sports Science and Medicine*.

[13] Sheppard A., Li F. X. (2007). Expertise and the control of interception in table tennis. *European Journal of Sport Science*.

[14] Bańkosz Z., Winiarski S., Malagoli L. I. (2020). Gender differences in kinematic parameters of topspin forehand and backhand in table tennis. *International Journal of Environmental Research and Public Health*.

[15] Sharif Bidabadi S., Murray I., Lee G. Y. F. (2018). Validation of foot pitch angle estimation using inertial measurement unit against marker-based optical 3D motion capture system. *Biomedical Engineering Letters*.

[16] Wu G., van der Helm F. C. T., Veeger H. E. J. D. J. (2005). ISB recommendation on definitions of joint coordinate systems of various joints for the reporting of human joint motion--part II: shoulder, elbow, wrist and hand. *Journal of Biomechanics*.

[17] Wu G., Siegler S., Allard P. (2002). ISB recommendation on definitions of joint coordinate system of various joints for the reporting of human joint motion--part I: ankle, hip, and spine. *Journal of Biomechanics*.

[18] Kontaxis A., Cutti A. G., Johnson G. R., Veeger H. E. J. (2009). A framework for the definition of standardized protocols for measuring upper-extremity kinematics. *Clinical Biomechanics*.

[19] Robinson M. A., Vanrenterghem J., Pataky T. C. (2021). Sample size estimation for biomechanical waveforms: current practice, recommendations and a comparison to discrete power analysis. *Journal of Biomechanics*.

[20] Friston K., Frackowiak R. S. J., Friston K. J., Frith C. D. (2004). *Experimental design and statistical parametric mapping*.

[21] Pataky T. C., Robinson M. A., Vanrenterghem J. (2013). Vector field statistical analysis of kinematic and force trajectories. *Journal of Biomechanics*.

[22] Pataky T. C. (2012). One-dimensional statistical parametric mapping in Python. *Computer Methods in Biomechanics and Biomedical Engineering*.

[23] Pataky T. C., Goulermas J. Y. (2008). Pedobarographic statistical parametric mapping (pSPM): a pixel-level approach to foot pressure image analysis. *Journal of Biomechanics*.

[24] Robinson M. A., Vanrenterghem J., Pataky T. C. (2015). Statistical parametric mapping (SPM) for alpha-based statistical analyses of multi-muscle EMG time-series. *Journal of Electromyography and Kinesiology*.

[25] Iino Y., Mori T., Kojima T. (2008). Contributions of upper limb rotations to racket velocity in table tennis backhands against topspin and backspin. *Journal of Sports Sciences*.

[26] Qian J., Zhang Y., Baker J. S., Gu Y. (2016). Effects of performance level on lower limb kinematics during table tennis forehand loop. *Acta of Bioengineering and Biomechanics*.

[27] Iino Y. (2018). Hip joint kinetics in the table tennis topspin forehand: relationship to racket velocity. *Journal of Sports Sciences*.

[28] Wang M., Fu L., Gu Y., Mei Q., Fu F., Fernandez J. (2018). Comparative study of kinematics and muscle activity between elite and amateur table tennis players during topspin loop against backspin movements. *Journal of Human Kinetics*.

[29] Yoichi I., Takeji K. (2016). Mechanical energy generation and transfer in the racket arm during table tennis topspin backhands. *Sports Biomechanics*.

[30] Marsan T., Rouch P., Thoreux P., Jacquet-Yquel R., Sauret C. (2019). Comparison of hip joint mechanical energetics in table tennis forehand and backhand drives. *International Journal of Racket Sports Science*.

[31] Petryński W. (2006). Topological tools in model of motor control in humans in Polish, Abstract in English Nnarzędzia topologiczne w opisie sterowania ruchami przez człowieka. *Antropomotoryka*.

[32] Xia R., Dai B., Fu W., Gu N., Wu Y. (2020). Kinematic comparisons of the shakehand and penhold grips in table tennis forehand and backhand strokes when returning topspin and backspin balls. *Journal of Sports Science and Medicine*.

